# Diagnosis of Cervical Intraepithelial Neoplasia and Invasive Cervical Carcinoma by Cervical Biopsy under Colposcopy and Analysis of Factors Influencing

**DOI:** 10.1155/2022/9621893

**Published:** 2022-07-30

**Authors:** Ying Wang, Jing Wang, Hua Mei

**Affiliations:** ^1^Medical Department of Wuhan Wudong Hospital, Wuhan 430084, Hubei, China; ^2^Hubei Materal and Child Health Hospital, Wuhan 430064, Hubei, China; ^3^Hospital Infection Branch, Wuhan Wudong Hospital Public Health, Wuhan 430084, Hubei, China

## Abstract

**Objective:**

To explore the diagnosis of cervical intraepithelial neoplasia (CIN) and invasive cervical carcinoma (ICC) by cervical biopsy under colposcopy and analyze the factors influencing the detection.

**Methods:**

The clinical data of 134 CIN confirmed by colposcopy biopsy in our hospital from June 2018 to October 2019 and subsequent LEEP treatment were analyzed retrospectively. All patients were diagnosed pathologically after the operation. The diagnosis of CIN by cervical biopsy under colposcopy was observed. The influencing factors of CIN and ICC detected by colposcopy biopsy were analyzed by the pathological results of loop electrosurgical excision procedure (LEEP) as the gold standard.

**Results:**

After LEEP, the number of the no intraepithelial or malignant lesions (NILM) or ICC were higher than that of colposcopy biopsy, and CIN-III was lower than that of colposcopy biopsy, the differences were all statistically significant (*P* < 0.05). Among the 134 patients, the coincidence rate between colposcopy biopsy and LEEP examination results was 79.10% (106/134), and postoperative pathological findings showed that there were 13 cases (9.70%) with the pathological upgrade and 19 cases (14.18%) with pathological decrease. Multivariate logistic analysis showed that the image quality of colposcopy image, atypical blood vessels, biopsy sampling method, and visible lesion area of the cervix were the independent influencing factors for the detection of CIN and ICC by colposcopy biopsy (*P* < 0.05).

**Conclusion:**

CIN and ICC can be diagnosed by colposcopy cervical biopsy and postoperative histopathology. However, there are still some missed and misdiagnosed cervical biopsies under colposcopy, and the combined detection of the two can further ensure the diagnosis rate. The clinical registration number is E2018091.

## 1. Introduction

Cervical cancer is a primary malignant tumor of the female reproductive system and is closely related to human papillomavirus, HPV) infection. In recent years, with the continuous promotion of early screening technology for cervical cancer, the early detection rate of cervical cancer increases year by year. However, its development shows a trend of younger people. Patients usually have unobservable early symptoms and signs. Stimulated by physicochemical and biological factors such as HPV infection and smoking, normal cervical cells will exhibit inflammatory and reactive changes, which can transition from the normal state to precancerous lesions, further develop into invasive cervical cancer, ICC), and finally develop into cervical cancer [1–3]. Cervical intraepithelial neoplasia (CIN) is the early manifestation of ICC, and its occurrence is diverse. It is a group of precancerous lesions closely related to the cancer process. CIN included cervical dysplasia and cervical carcinoma in situ, reflecting a series of pathological changes from cervical dysplasia, carcinoma in situ, and early invasive carcinoma to invasive carcinoma. CIN can be diagnosed through cytology, colposcopy, and other examinations [4–6]. Among them, cervical biopsy under colposcopy is a common tissue examination method for the diagnosis of CIN, and it refers to observing the state of precancerous lesions of tissues with the help of a colposcope and taking the corresponding tissues for pathological examination [7, 8]. However, due to the complexity and diversity of CIN and the unclear classification, the effect of CIN by colposcopy cervical biopsy is not very accurate and it is easy to cause a certain misdiagnosis or missed diagnosis. Therefore, in this study, we investigated the diagnosis of CIN and ICC by colposcopy cervical biopsy and analyzed the effects of relevant factors on the detection.

## 2. Materials and Methods

### 2.1. General Information

The clinical data of 134 patients who were diagnosed as CIN by colposcopy biopsy and subsequently treated with Loop Electrosurgical Excision Procedure (LEEP) from June 2018 to October 2019 in our gynecological clinic were analyzed retrospectively. All the patients were aged from 20 to 52 years old, with an average age of (36.52 ± 3.26) years old. Inclusion criteria: Inclusion criteria: Contact bleeding, irregular vaginal bleeding, abnormal drainage, and other symptoms; Meet the indications of colposcopy; HPV-DNA test positive; Abnormal cervical cytology. Exclusion criteria: Mental disorder; Low compliance, unable to cooperate with the inspection; In pregnancy; Important organ dysfunction.

### 2.2. Research Method

#### 2.2.1. Detection of Cervical Cytology

A sterile sampling brush was placed into the cervical canal and rotated 5–10 times to collect the exfoliated cells from the cervical external orifice and the canal, which were then put into a bottle containing the preservation solution. The samples were sent for inspection after being washed ≥10 times and processed by a slide maker. Two pathologists in the hospital performed light microscopic diagnosis and cytological results were processed. The cytological results were divided into the advanced lesion group and conventional lesion group according to The Bethesda System (TBS). TBS includes five types according to the degree of cervical cell lesions. We divide them into advanced lesion groups and conventional lesion groups according to the degree of cervical cell lesions [9]. The advanced lesion group included atypical squamous cell hyperplasia (ASCH), high-grade intraepithelial lesions (HSIL), and ICC. The conventional lesion group included no intraepithelial or malignant lesions (NILM), atypical squamous cells of undetermined significance (ASCUS), and low-grade squamous intraepithelial lesions (LSIL).

#### 2.2.2. Detection of High-Risk HPV (HR-HPV)

The cervix was exposed through the vaginal endoscope. After the secretion on the surface of the cervical orifice was wiped, a sterile cotton swab was inserted into the cervix and rotated around the interior of the cervix three times with uniform force. Afterward, the swab was taken out and put into a sample storage box for submission. Samples were quantified by fluorescent PCR typing and an HR-HPV viral load > 5.0 × 102 copies/mL was defined as positive. HR- HPV mainly includes 15 kinds of HPV16, 18, 31, 33, 35, 39, 45, 51, 52, 56, 58, 59, 68, 73, 82, and so on. a total of 49 cases of HPV16, 15 cases of HPV26 and 10 cases of other types were detected in this test.

#### 2.2.3. Colposcopic Biopsy

All patients had no sexual activity, vaginal medication, or any gynecological examination within 24 hours, and samples were taken during the nonmenstrual period and genital tract infection period. Processing pictures by adopting an electronic colposcope digital imaging system; The patient was told to keep the cystectomy position, and the color, morphology, secretion, and leukoplakia of the cervix were observed by the naked eye. According to the different patients, the appropriate endoscope was used for examination. The cervix of the patient was fully exposed under the endoscope, and the surface of the cervix was gently wiped with a medical cotton swab to remove the foreign body. After the removal of the foreign body, normal saline was uniformly applied to the cervix. Then, the colposcope was adjusted to focus the lens, and the junction of the epithelium and blood vessel by the scale column was observed. Apply 3% acetic acid to the cervix, and carefully observe the abnormal angiogenesis and columnar epithelial edema of the cervix. The Lugol's iodine solution was applied to the cervix to observe the epithelial staining. And single-point or multi-point sampling biopsy was conducted for the abnormal parts. If no abnormality is found, the lower four-quadrant sampling biopsy will be conducted.

#### 2.2.4. LEEP

Preoperative patients were required to empty the bladder and take the lithotomy position of the bladder. After routine disinfection, the cervix of the patient was fully exposed. According to the patient's history and clinical symptoms, and iodine staining test was performed on the cervical lesion site of the patient under a colposcope to determine the lesion site of the patient. The LEEP knife was reasonably selected according to the lesion area and cervix size of the patient. The electrodes were vertically cut into the cervical tissue from the external source of the lesion for 5–6 mm, and the depth was controlled to be about 1.0–2.5 cm for resection, followed by marking, positioning, fixation, and submission of the specimen.

Tissue samples of all patients were pathologically reviewed by two attending physicians of the Department of Pathology and classified into NILM, mild atypical hyperplasia (CIN-I), moderate atypical hyperplasia (CIN-II), severe atypical hyperplasia (CIN-III) and ICC according to CIN classification standard [10]. NILM: HPV infection was negative, the epithelium showed inflammatory cell infiltration reaction, and no obvious lesion area was observed. CIN-I: The epithelial cells are featured with mild atypia, disordered polarity, and abnormal proliferation, accounting for 1/3 of the subcortical range of the upper cortex. CIN-II: The epithelial cells are heterotypic and disorganized, and abnormally proliferate to two-thirds of the subcortical range of the upper cortex. CIN-III: The epithelial cells are heterotypic and nonpolar, with abnormal proliferation (>2/3 of the subepithelial range) and no interstitial infiltration. ICC: Abnormal proliferation of epithelial cells involving the entire epithelial layer, with pathological mitosis and interstitial infiltration. The highest grade of histological diagnosis was the final pathological examination in all patients.

### 2.3. Statistical Analysis

SPSS22.0 software was used for data processing. The count data were expressed as (%) using the *χ*^2^ test. A multivariate Logistic regression model was used for multivariate analysis. The test level was *α* = 0.05, and *P* < 0.05 indicated that the difference was statistically significant.

## 3. Results

### 3.1. Comparison of Pathological Examination Results after Colposcopic Biopsy and LEEP

The numbers of NILM and ICC cases after LEEP operation were higher than those of colposcopy biopsy, and the number of CIN-III cases was lower than that of colposcopy biopsy. The differences were statistically significant (*P* < 0.05). Among the 134 patients, the coincidence rate between colposcopy biopsy and LEEP examination results was 79.10% (106/134), and postoperative pathological findings showed that there were 13 cases (9.70%) with the pathological upgrade and 19 cases (14.18%) with pathological decrease. See Figure 1.

### 3.2. Single Factor Analysis of Influencing the Detection of CIN and ICC in Colposcopic Biopsy

Univariate analysis showed that patients with age ≤ 50 years old, satisfactory colposcopic image, atypical blood vessels, four-quadrant biopsy sampling method, number of biopsy samples >2, visible lesion area of cervix ≥1/2, and pathological grade (CIN-III/invasive cervical cancer) had high detection rates of CIN and ICC under colposcopy, and the differences were statistically significant (both *Ps* < 0.05). The detection rates of CIN and ICC in cytology tests and HR-HPV infection were not statistically significant (*P* > 0.05). See Table 1.

### 3.3. Multivariate Analysis of Influencing Factors on Detection of CIN and ICC in Colposcopic Biopsy

Multivariate Logistic analysis showed that the image quality of colposcopic image, atypical blood vessels, biopsy sampling method, and visible lesion area of the cervix was the independent influencing factors for the detection of CIN and ICC by colposcopy biopsy (*P* < 0.05); see Tables 2 and 3.

## 4. Discussion

The pathological types of cervical cancer mainly include squamous cell carcinoma, adenocarcinoma, and adenosquamous carcinoma. The pathological change and development process of various types of cervical cancer are closely related to many factors, such as virus infection, bad living habits, and so on, which cause serious impacts on the physical life of women. Cervical cancer has now become the “second largest killer” threatening women s health after breast cancer [11]. Therefore, early screening, early detection, early diagnosis, and early treatment of cervical cancer are particularly important. CIN is an important pathological stage before the occurrence of cervical cancer, which is usually manifested as irregular vaginal bleeding, increased leucorrhea, and unpleasant odor. The incidence rate of patients is high and it has certain concealment. Early detection, diagnosis, and treatment of CIN are conducive to interfering with the lesion progression and reducing the incidence of cervical cancer [12].

Cervical biopsy under colposcopy is a technical means for clinical promotion and application of diagnosis of CIN. However, under the magnification of colposcopy, clinicians can identify the lesion area with the naked eye, and conduct biopsy sampling accidentally or blindly, so there are problems of high sensitivity and low specificity. LEEP is an advanced technical means for the treatment of various cervical lesions, which mainly generates thermal effect through ohmic consumption of high-frequency current through the human body, to evaporate the water in the tissue, achieving the effects of dry solid, sterile necrosis [13]. There is a certain error between the accuracy of colposcopic cervical biopsy and the pathological diagnosis after LEEP surgery, and the pathological grade may be increased or decreased [14, 15]. The results of this study showed that the numbers of NILM and ICC cases after LEEP operation were higher than those of colposcopic biopsy, and the number of CIN-III cases was lower than that of colposcopic biopsy. Among 134 patients, the coincidence rate of colposcopic biopsy and postoperative pathological examination results of LEEP was 79.10%, and postoperative pathological findings showed that there were 13 cases (9.70%) with the pathological upgrade and 19 cases (14.18%) with pathological decrease. This result was partially consistent with that of Zhang et al. [16].

ICC is not only a clinical manifestation of high-risk CIN but also an early pathological manifestation of cervical cancer. Because the process of differentiation and expression of cancer cells are very disorderly, the abnormal expression of vascular endothelial genes can lead to invasive invasion of cancer cells and diversified expression of cancer markers, which will cause certain difficulties in direct vision and pathological film reading [17–19]. Many studies have shown that the diagnostic rate of ICC colposcopic cervical biopsy remains to be improved, and its detection rate is affected by many factors, such as the number of lesion-involved points [20, 21]. Therefore, exploring the influencing factors of the accuracy of the cervical biopsy under colposcopy is of great significance for improving the detection rate of ICC. The univariate analysis of this study showed that the detection rates of CIN and ICC in the colposcopic cervical biopsy were related to the patient's age, colposcopic image, presence of atypical blood vessels, sampling method, and several biopsy samples, visible lesion area of cervix and pathological grade. The colposcopic image, presence of atypical blood vessels, sampling method of biopsy, and visible lesion area of the cervix were the independent influencing factors for their detection. The possible reason for this analysis was that there was a certain difference in the image quality under colposcopy, which affected the directness of the lesion site and further caused the corresponding deviation of endoscopic sampling. Therefore, continuous improvement of the image quality under colposcopy and the direct visualization of cervical lesions as well as the adoption of sampling methods such as multi-quadrant biopsy can help to reduce the missed diagnosis and misdiagnosis rate of the cervical biopsy under colposcopy in clinical practice [22].

In summary, CIN and ICC can be diagnosed by colposcopic cervical biopsy and postoperative histopathological examination. However, there are still some missed diagnoses and misdiagnoses in cervical biopsy under colposcopy, and the combined detection of the two can further ensure the diagnosis rate.

## Figures and Tables

**Figure 1:** Comparison of pathological examination results after colposcopic biopsy and LEEP operation.

**Table 1:** Single-factor analysis of influencing the detection of CIN and ICC in the colposcopic biopsy.

Influencing factor		Case (*n* = 134)	Number of detected cases	Number of missed cases	Detection rate (%)	*χ* ^*2*^ value	*P* Value
Age (year)	≤50	84	72	12	85.71	4.811	0.028
	>50	50	35	15	70.00		
Cytological test	Advanced lesion group	79	47	32	59.49	3.259	0.071
	Conventional lesion group	55	41	14	74.55		
Infection of HR-HPV	Negative	52	45	7	86.54	3.353	0.067
	Positive	82	60	22	73.17		
Colposcopic image	Satisfied	58	44	14	75.86	5.371	0.020
	Dissatisfied	76	43	33	56.58		
Atypical blood vessel	Yes	52	41	11	78.85	4.663	0.031
	No	82	50	32	60.98		
Biopsy sampling method	Four quadrant sampling	65	57	8	87.69	6.485	0.011
	Single/multiple point lesion sampling	69	48	21	69.57		
Number of biopsy sample (s)	≤2	64	43	21	67.19	4.423	0.035
	＞2	70	58	12	82.86		
Visible lesion area of the cervix	＜1/2	65	40	25	61.54	5.356	0.021
	≥1/2	69	55	14	79.71		
Pathological grade	NILM/CIN-I∼II	63	39	24	61.90	3.860	0.049
	CIN-III/ICC	71	55	16	77.46		

**Table 2:** Multivariate analysis of the assignment.

Influencing factor	Assignment
Age	“>50” = 0; “≤50” = 1
Colposcopic image	“Dissatisfied” = 0; “satisfied” = 1
Atypical blood vessel	“No” = 0; “yes” = 1
Biopsy sampling method	“Single/multiple point lesion sampling” = 0; “four quadrant sampling” = 1
Number of biopsy sample (s)	“≤50” = 0; “>50” = 1
Visible lesion area of the cervix	“≤2” = 0; “>2” = 1
Pathological grade	“≤1/2” = 0; “≥1/2” = 1

**Table 3:** Multivariate analysis of influencing factors on detection of CIN and ICC in the colposcopic biopsy.

Influencing factor	*B*	*SE*	*Walds*	df	Sig.	Exp (B)	95% CI
Age	0.279	0.184	2.958	1	0.064	1.639	0.978∼2.316
Colposcopic image	0.656	0.227	5.133	1	0.029	2.374	1.786∼2.997
Atypical blood vessel	0.712	0.256	5.266	1	0.016	2.241	1.853∼2.761
Biopsy sampling method	0.754	0.343	5.307	1	0.009	2.580	2.042∼3.159
Number of biopsy sample (s)	0.305	0.229	3.164	1	0.056	2.475	0.768∼2.991
Visible lesion area of the cervix	0.816	0.387	4.644	1	0.032	2.837	1.911∼3.796
Pathological grade	0.263	0.152	2.548	1	0.120	1.532	0.733∼2.910

## Data Availability

The datasets generated during and/or analyzed during the current study are available from the corresponding author on reasonable request.

## References

[1] Temkin S. M., Rimel B. J., Bruegl A. S., Gunderson C. C., Beavis A. L., Doll K. M. (2018). A contemporary framework of health equity applied to gynecologic cancer care: a society of gynecologic oncology evidenced-based review. *Gynecologic Oncology*.

[2] Pimple S. A., Mishra G. A. (2019). Global strategies for cervical cancer prevention and screening. *Minerva Ginecologica*.

[3] Saleh M., Virarkar M., Javadi S., Elsherif S. B., de Castro Faria S., Bhosale P. (2020). Cervical cancer: 2018 revised international federation of gynecology and obstetrics staging system and the role of imaging. *American Journal of Roentgenology*.

[4] Bui C. N., Hong S., Suh M. (2021). Effect of pap smear screening on cervical cancer stage at diagnosis: results from the Korean national cancer screening program. *Journal of Gynecologic Oncology*.

[5] Allanson E. R., Schmeler K. M. (2021). Preventing cervical cancer globally: are we making progress?. *Cancer Prevention Research*.

[6] Wilailak S., Kengsakul M., Kehoe S. (2021). Worldwide initiatives to eliminate cervical cancer. *International Journal of Gynecology & Obstetrics*.

[7] Rajaram S., Gupta B. (2022). Screening for cervical cancer: choices & dilemmas. *Indian Journal of Medical Research*.

[8] Alder S., Megyessi D., Sundström K. (2020). Incomplete excision of cervical intraepithelial neoplasia as a predictor of the risk of recurrent disease-a 16-year follow-up study. *American Journal of Obstetrics and Gynecology*.

[9] Baloch Z., LiVolsi V. A. (2020). The Bethesda system for reporting thyroid cytology (TBSRTC): from look-backs to look-ahead. *Diagnostic Cytopathology*.

[10] Horn L. C., Beckmann M. W., Follmann M. (2015). S3 guidelines on diagnostics and treatment of cervical cancer: demands on pathology. *Der, Pathologe*.

[11] Grimm D., Lang I., Prieske K. (2020). Course of cervical intraepithelial neoplasia diagnosed during pregnancy. *Archives of Gynecology and Obstetrics*.

[12] Burki T. K. (2019). Therapeutic HPV vaccine for cervical intraepithelial neoplasia. *The Lancet Oncology*.

[13] Parajuli G., Dawadi P., Khadka S. (2020). Prevalence of cervical cancer among cervical biopsies in a tertiary care center. *JNMA: Journal of the Nepal Medical Association*.

[14] Gabrielli S., Maggioni E., Fieschi L. (2018). Cervical cancer prevention in Senegal: an international cooperation project report. *Acta BioMedica*.

[15] Chang H. K., Seo S. S., Myong J. P., Yu Y. L., Byun S. W. (2019). Incidence and costs of cervical intraepithelial neoplasia in the Korean population. *Journal of Gynecologic Oncology*.

[16] Zhang H., Xiao J. N., Tao X., Zhou X. R., Wang L. (2018). Consistency of diagnosis between cervical cytology and colposcopic biopsy diagnosis. *Zhonghua Bing Li Xue Za Zhi*.

[17] Agarwal P., Bakshi P., Verma K. (2021). Liquid-based cytology of amoebic cervicitis clinically mimicking cervical cancer. *Diagnostic Cytopathology*.

[18] Shimada C., Todo Y., Yamazaki H., Minobe S., Kato H. (2019). Cervical laser vaporization for women with cervical intraepithelial neoplasia-3. *Japanese Journal of Clinical Oncology*.

[19] Hoffman S. R., Le T., Lockhart A. (2017). Patterns of persistent HPV infection after treatment for cervical intraepithelial neoplasia (CIN): a systematic review. *International Journal of Cancer*.

[20] Curty G., de Carvalho P. S., Soares M. A. (2019). The role of the cervicovaginal microbiome on the genesis and as a biomarker of premalignant cervical intraepithelial neoplasia and invasive cervical cancer. *International Journal of Molecular Sciences*.

[21] Kalliala I., Athanasiou A., Veroniki A. A. (2020). Incidence and mortality from cervical cancer and other malignancies after treatment of cervical intraepithelial neoplasia: a systematic review and meta-analysis of the literature. *Annals of Oncology*.

[22] Øvestad I. T., Engesæter B., Halle M. K. (2021). High-grade cervical intraepithelial neoplasia (CIN) associates with increased proliferation and attenuated immune signaling. *International Journal of Molecular Sciences*.

